The article "Deep Fusion of Intelligent Meridian Sensing Technology and Huoluo Xiaoling Pills in the Treatment of Knee Osteoarthritis" was retracted in 2023. Reasons: signs of a paper mill; suspected computer-generated content; unreliable results or conclusions; concerns about the data.

# Deep Fusion of Intelligent Meridian Sensing Technology and Huoluo Xiaoling Pills in the Treatment of Knee Osteoarthritis

**DOI:** 10.1155/2022/8043674

**Published:** 2022-09-07

**Authors:** Jiye Sun, Ziou Wang, Piao Wu, Jinxuan Wei, Xiaowei Sun, Hongtao Li

**Affiliations:** ^1^Heilongjiang University of Chinese Medicine, Harbin 150000, China; ^2^The First Affiliated Hospital of Heilongjiang University of Chinese Medicine, Harbin 150000, China

## Abstract

Based on the deep fusion of intelligent meridian sensing technology and Huoluo Xiaoling Pill (HXP) in the treatment of knee osteoarthritis (KOA), firstly, the effective components and targets of *Salvia miltiorrhiza*, *Angelica sinensis*, *frankincense*, and *myrrh* were obtained by using TCMSP, SwissADME, and Swisstarget databases. Similarly, relevant targets of KOA were collected through GeneCards, OMIM, TTD, PharmGKB, and DrugBank databases. Next, the potential targets of ZXP in the treatment of KOA were obtained by intersection of drug and disease targets. Finally, Cytoscape 3.7.1 software was used to construct a “disease-drug-component-target” network, and Gene Ontology (GO) function and Kyoto Encyclopedia of Genes and Gnomes (KEGG) signaling pathway enrichment analysis were performed on the core targets through Metascape website. A total of 99 active components and 203 corresponding potential therapeutic targets were obtained from the components of HXP. And KOA has 2543 potential therapeutic targets, of which 120 cross targets correspond to 120 active compounds in HXP. Then, topology analysis displayed that the six targets form the core PPI network. In addition, GO and KEGG enrichment analyses showed that these core targets were mainly enriched in inflammatory response, apoptosis, oxidation reaction, and other related pathways.

## 1. Introduction

Knee osteoarthritis (KOA), belonging to the category of osteoarthritis (OA), is a common disease with continuous knee pain, morning stiffness, limited activity, and reduced function [1]. The specific etiology of the disease is not yet clear. At present, it is mainly believed that the disease is caused by the interaction of factors such as heredity, age, and hormone deficiency [2]. In the world, OA is the most common adult joint disease [3], of which KOA is the most common type, accounting for about 6% of all adults [4]. In China, the incidence rate of KOA is 18%, and significantly, the prevalence of female is higher than male, which affects the quality of life of patients and causes a certain economic burden seriously [5]. At present, the recognized clinical treatment methods for KOA mainly include patient education, physical therapy, NSAIDs, knee repair, and reconstruction [6].

KOA that belongs to the category of “bone arthralgia disease” and “knee arthralgia disease” in traditional Chinese medicine (TCM) can be divided into cold dampness arthralgia, damp heat arthralgia, qi stagnation and blood stasis, liver and kidney deficiency, and qi and blood weakness [7]. Acupuncture, moxibustion, massage, herbal medicine, and other TCM treatments can affect relevant signaling pathways and then inhibit knee inflammation through a variety of noninvasive or minimally invasive treatments to alleviate pain. At the same time, it can avoid the side effects of relevant western medicine treatments and the abuse of analgesic drugs.

Huoluo Xiaoling Pill (HXP) is used for promoting blood circulation and removing blood stasis, dredging meridians and relieving pain, treating qi and blood stasis, confidant pain, leg and arm pain, etc. There were frequent additions and subtractions in orthopaedic therapy for closed fractures, compartment syndrome (OFCS), traumatic knee synovitis combined, and so in [8]. Additionally, modern medical research shows that HXP has pharmacological reactions of anti-inflammatory, detumescence, and analgesia, which can effectively promote the regression of edema, relieve tissue compression, and improve local microcirculation [9]. In 2007, the British pharmacologist Hopkins first proposed the concept “network pharmacology” that has been widely used in clinical and pharmacological research [10], so as to further clarify the action pathway and mechanism of traditional Chinese medicine and provide a theoretical basis for the efficacy and efficacy of traditional Chinese medicine [11]. Schütze et al. highlight some of the potential that smart sensors and data evaluation can achieve and discuss the requirements for success in future development, discussing condition monitoring as the main paradigm for the introduction of smart sensors and data analytics in manufacturing-based processes in two of their projects in [12]. Mohammed et al. propose an IoT device and sensor management framework for smart medical solutions. This framework is designed to be integrated into electronic health gateways and patient intelligence devices and accessories [13]. Zhu et al. discussed different aspects of smart healthcare and health data and patient-centred health management [14, 15].

In this study, the treatment of KOA by HXP was analyzed by NP, which provided direction and enlightenment for exploring the drug action mechanism of HXP. This study is aimed at exploring the potential mechanism of HXP in the treatment of KOA through the method network pharmacology (NP), which may contribute to the screening of clinical drugs for KOA and improve the dosage form of HXP, providing reference for exploring the matrix of HXP in the treatment of KOA.

## 2. Materials and Methods

The intelligent meridian therapy instrument is guided by the basic theory of traditional Chinese medicine. The dynamic interference frequency conversion pulse therapy used is based on the traditional acupuncture theory, which combines high voltage and low frequency conversion pulses with the meridian theory. The internal and external knee eye points) are electrically stimulated to achieve the day of clearing the meridians, promoting blood circulation and removing blood stasis, promoting qi, and relieving pain. Meridian physiotherapy instrument can play a role in adjuvant treatment and remission for some inflammatory diseases and can assist in the treatment of some nervous system diseases.

### 2.1. Acquisition of HXP Active Components and Targets Screening

The chemical components of *Salvia miltiorrhiza* (Dan Shen in Chinese), *Angelica sinensis* (Dang Gui in Chinese), *frankincense* (Ru Xiang in Chinese), and *myrrh* (Mo Yao in Chinese) in HXP were obtained by TCMSP database (Traditional Chinese Medicine Systems Pharmacology, (https://tcmspw.com/tcmsp.php). Further, the effective components and target information, which were obtained in virtue of screening according to the restrictions of drug oral bioavailability (OB) ≥ 30% and drug like (DL) ≥ 0.18%, convert the obtained target information into the verified human gene identification code in UniProt database (https://www.uniprot.org/) for subsequent use.

### 2.2. Screening of Disease Targets in KOA

“Knee osteoarthritis,” “knee arthritis of knees,” and “knee arthritis in the knee” were entered into DrugBank (https://go.drugbank.com/), GeneCards, OMIM (Online Mendelian Inheritance in Man, (https://omim.org/), TTD (Therapeutic Target Database, http://bidd.nus.edu.sg/group/cjttd/), and PharmGKB databases (https://www.pharmgkb.org/) to search for disease targets related to KOA, respectively. After all results were screened and deduplicated, target information of KOA was obtained.

### 2.3. Screening of Common Targets of Drugs and Diseases

The common targets of drugs and diseases are obtained through the pug(a process of writing code by indenting) in the R Programming Language (R), and the Venn diagram (Venn) is drawn. Drug targets refer to the binding sites of drugs in the body, including biological macromolecules such as genetic loci, receptors, enzymes, ion channels, and nucleic acids.

### 2.4. Construct the “Drug-Component-Target-Disease” Network Model

The active components of drugs obtained by “1.2.1,” common targets of drug diseases gained by “1.2.3,” and the network information between them are imported into Cytoscape 3.7.1 to construct the network diagram. Each node is the target, component, and drug name, respectively, between which each edge represents the interaction relationship.

### 2.5. Construct Protein-Protein Interaction (PPI) Network

The common targets of drug diseases obtained in “1.2.3” are imported into STRING database, and the species is limited to human, to obtain PPI information, which is imported into the Cytoscape 3.7.1 to generate PPI network diagram, and then, the CytoNCA plug-in is used to conduct topological analysis on the network data. First of all, the degree centrality (DC) nodes which are greater than twice median are screened. After that, the index parameters of betweenness, closeness, local average connection-based method (LAC), and neighborhood connectivity were greater than the twofold median. Eventually, the core targets of HXP in the treatment of KOA were obtained, and the PPI core network was mapped. The interaction between proteins is the basis for the occurrence of life phenomena, and the study of their interactions can clarify the mechanism of biological reactions and reveal the essence of life phenomena.

### 2.6. GO and KEGG Enrichment Analyses

First, add 1.2.3, the obtained intersection targets were introduced into the Metascape, and human species were selected. Afterwards, the GO and KEGG enrichment analyses were carried out separately under the limiting conditions of minimum overlap of 3, *P* < 0.01, and minimum enrichment of 1.5, the GO analysis of which also includes the data analysis of biological process (BP), molecular function (MF), and cellular component (CC). In the end, the top 10 items obtained from GO-BP, GO-MF, and GO-CC and the first 20 results from KEGG were selected, respectively, being drawn into bubble chart for visual processing via origin Lab 2018. The size of bubble represents the number of targets enriched in the specified path, while the color means the enriched *q* value. As shown in Figure 1.

## 3. Results

### 3.1. Screening of Active Components and Targets

A total of 99 effective components of HXP were obtained, including 59 *Salvia miltiorrhiza*, 2 *Angelica sinensis*, 6 *frankincense*, and 34 *myrrh*, where *Angelica sinensis* and *myrrh* also contain *β*-sitosterol and stigmasterol (Table 1). The active ingredients include luteolin, sugiol, isoimperatorin, and poriferast-5-en-3beta-ol. Beyond that, the 1285 targets converted from the UniProt were deduplicated, acquiring 203 target information such as ptgs1, ADRB2, ESR2, and MMP1.

### 3.2. Screening of Disease Targets

Taking “knee osteoarthritis,” “osteoarthritis of knees,” and “osteoarthritis in the knee” as keywords, the target information obtained from multiple databases was screened and deduplicated, where a total of 2543 disease-related targets were acquired, there being 71 DrugBank, 2292 GeneCards, 228 OMIM, 9 PharmGKB, and 1 TTD among them. Through the integrated analysis of high-throughput omics data from multiple levels and sources, systematically studying the clinical pathogenesis and determining the best disease targets have become an important development direction of precision medicine research, which will provide new ideas for disease research. It also provides a new theoretical basis for the early diagnosis of the disease, individualized treatment, and guidance of medication.

### 3.3. Screening of Common Targets of Drugs and Diseases

The 203 drug targets in “2.1” and 2543 disease targets in “2.2” were processed by R-Venn to obtain a total of 120 drug-disease common targets (Figure 2).

### 3.4. Construction of “Drug-Component-Target-Disease” Network Model

The 99 active components of HXP and drug-disease common targets were introduced into the Cytoscape to generate a “drug-component-target-disease” network model (Figure 3), which includes 214 nodes (4 drug name nodes, 120 target nodes, and 90 active ingredient nodes) and 759 edges (93 drug and active ingredient connections and 666 active ingredient and target connections). Nine active ingredients without related targets are deleted, and 28 components with connectivity not less than 10 among the 90 active ingredients in Figure 3 are listed in Table 2, including quercetin, luteolin, *β*-sitosterol, tanshinone IIA, and dihydrotanshinlactone having a larger degree of connectivity, which means that they play a more extensive role.

### 3.5. Construction of PPI Network and Screening of Core Targets

The common drug-disease targets obtained in 2.3 were imported into the STRING to construct PPI network, as shown in Figure 4 (left). And 120 targets and 4316 edges of interaction were acquired, and the results were introduced into the Cytoscape. In addition, CytoNCA plug-in is used to conduct network analysis and screen the nodes whose values of betweenness, closeness, degree, LAC, and neighborhood connectivity are greater than twice the median to get the core network that includes 5 core targets (STAT1, RELA, NFKBIA, BCL2L1, HMOX1, and MAPK14) and 28 interrelations, suggesting that these targets may play a key role in the treatment of KOA with HXP, as shown in Figure 4 (right).

### 3.6. GO Enrichment Analysis

The so-called enrichment analysis is essentially a test of the distribution. If the distribution is concentrated in a certain area, it is considered enriched. The 120 drug-disease common targets obtained in 2.3 were enriched and analyzed by the Metascape to get GO items that meet the screening conditions, from which the first 10 pathways of BP, CC, and MF in GO items were selected for bubble chart (Figures 5–7); the results show that the BP of HXP for the treatment of KOA mainly involved the response to organic matter, radiation, and lipopolysaccharide; the CC mainly involved membrane raft, cytoplasmic perinuclear region, transcriptional regulatory complex, and so on; the MF mainly involved transcription factor binding, protein kinase binding, mucus receptor activity, etc.

### 3.7. KEGG Enrichment Analysis

KEGG enrichment analysis was performed on the Metascape for 120 drug-disease common targets obtained in 2.3, and 150 KEGG items meeting screening conditions were acquired, the top 20 ways of which were selected for bubble chart (Figure 8), displaying that the main signaling pathways involved in the treatment of KOA by HXP were signal transduction (IL-17; AGE-RAGE, HIF-1, P53, NF-*κ*B, estrogen, prolactin, MAPK, JAK-STAT, and VEGF signals in diabetic complications), viral and parasitic infections (hepatitis B virus, malaria, prions, and amoebiasis), cancer and transcriptional disorders in cancer, nonalcoholic fatty liver disease, rheumatoid arthritis, etc. According to the comparison between the core targets gained in 2.5 and the genes obtained by each KEGG pathway, 32 pathways related to KOA were selected through comparison with the existing literature, and the top 20 pathways with larger enrichment factors were chosen for display (Table 3), among which IL-17 signaling pathway, TNF signaling pathway, PI3K-Akt signaling pathway, etc. were enriched with more genes and higher enrichment factors. A kind of preinflammatory cytokines secreted by CD4^+^ T cells can induce the release of inflammatory factors, which plays an important role in both acute and chronic inflammatory reactions, and can destroy the balance between osteogenesis and osteoclast in KOA, which aggravates the destruction of cartilage tissue.

## 4. Discussion

Intelligent medical care is to realize the interaction between patients and medical staff, medical institutions, and medical equipment by building a regional medical information platform for health records and using the most advanced Internet of Things technology and gradually achieve informatization. In the near future, the medical industry will incorporate more high-tech technologies such as artificial intelligence and sensing technology, so that medical services will become truly intelligent and promote the prosperity and development of the medical industry. In the context of China's new medical reform, intelligent medical care is entering the lives of ordinary people.

The architecture of wireless sensor network healthcare system generally consists of three parts. The first part is the monitoring object; it refers to the elderly and the environment in which the elderly live; the second part is the nursing staff. Nursing staff include remote service centers, doctors, nurses, and relatives of the elderly; the third part is access equipment, including public communication networks (PCNs) and gateways.

This study explored the potential targets and mechanism of HXP in the treatment of KOA through NP. The 99 drug active ingredients and 120 intersection targets obtained were used to construct the “drug-component-target-disease” network model, and the analysis showed that most of the ingredients affected multiple targets. For example, quercetin, luteolin, beta-sitosterol, tanshinone IIA, and dihydrotanshinlactone have affected 90, 44, 32, 24, and 17 targets, respectively, so they may be the most concernful active components of HXP. Quercetin and, at the same time, multiple active components can act on the same target, which proves that these have synergistic effects on the target. Quercetin belongs to flavonol and is one of the six subclasses of flavonoids and has anticancer, anti-inflammatory, and antiviral activities, as well as the effects of reducing lipid peroxidation, platelet aggregation, and capillary permeability [12], which have be shown by studies. For KOA, it can eliminate knee cartilage degradation and reduce chondrocyte apoptosis through antioxidant and anti-inflammatory [13]. Additionally, plants rich in luteolin, a common flavonoid, have been used to treat various diseases, such as hypertension, inflammation, and cancer [14, 15]. Fei et al. have proved that luteolin has anti-inflammatory effect on chondrocytes by treating these cells with different concentrations of it [16]. What is more, *β*-sitosterol, an antioxidant [17], is widely used in the treatment of atherosclerosis, diabetes, cancer, and inflammation. By analyzing the active components of many drugs with high oral availability and connectivity, it is considered that the therapeutic effect of HXP on KOA may be through anti-inflammatory, inhibiting osteoclast and apoptosis.

Through the analysis of the core network, some information that may be helpful to explain the effect of HXP is also explained. NFKBIA, NF-*κ*B inhibitor *α*, is an important inhibitor of NF-*κ*B that binds to the NF-*κ*B complex and further inactivates NF-*κ*B by retaining its cytoplasmic localization, which has been proved to promote the development of OA by promoting inflammation, stress, and chondrocyte hypertrophy differentiation [18]. And RELA, a key subunit mediating NF-*κ*B signaling, is involved in cartilage formation and differentiation, cell survival, and the production of catabolic enzymes, which exerts antiapoptotic effects on chondrocytes during bone growth and articular cartilage homeostasis [19]. Besides, heme oxygenase 1 (HMOX1) showed cytoprotective effects by cutting heme and reducing its content to reduce the sensitivity of cells to apoptosis, which were antioxidant, antiapoptotic, and anti-inflammatory [20]. Moreover, BCL2L1, a potent inhibitor of apoptosis, alleviates the development of KOA by inhibiting apoptosis. The results of core network analysis can also reveal the internal mechanism of HXP in the treatment of KOA from the main targets, so as to verify its effectiveness.

Go and KEGG analyses further verified the above, especially KEGG analysis, which displayed that IL-17 and TNF were the pathways with high enrichment factors and genes. At present, the research on KOA has found that its pathological and physiological process mainly includes the catabolism mediated by inflammatory cytokines and other mediators, as well as the protective effect of anti-inflammatory cytokines on joint tissue [21]. IL-17 is a key mediator of inflammation, and through its synergy with other inflammatory signals, it has become an important effector to examine inflammation [22], Its mediated activation of PI3K/Akt/mTOR resulted in down-regulation of cirs-7 and up-regulation of miR-7, aggravated cartilage degeneration and autophagy [23]. And TNF, as an immunological central modulator, is the core of host defense and inflammatory response, basically mediating inflammatory response, tissue degeneration, immune regulation, and tissue regeneration [24, 25]. Further analysis of related pathways indicated that the treatment of KOA by HXP may be mediated by these pathways to regulate the reactions such as inflammation, tissue degeneration and regeneration, apoptosis, autophagy, etc.

*Angelica sinensis* and *Salvia miltiorrhiza* in the prescription can quicken the blood and dispel stasis and free collaterals vessels and relieve pain; *frankincense* and *myrrh* are commonly used in traumatology to quicken the blood and free collaterals vessels and dispel stasis and relieve pain. For KOA, the whole prescription plays the functions of quickening the blood and removing stasis and freeing collaterals vessels and relieving pain. The above network pharmacological analysis of HXP also coincides with the traditional Chinese medicine theory of the action mechanism of HXP drugs. Although all drugs play different roles in the treatment of KOA, most of the components with high connectivity come from *Salvia miltiorrhiza*, and the traditional Chinese medicine theory will also take *Salvia miltiorrhiza*, which plays a strong role, as the king medicine of this prescription. The unification of these two theoretical verification results not only provides more favorable evidence for the action mechanism of HXP but also provides new ideas for the follow-up drug research and development.

KOA belongs to “knee arthralgia disease” and “bone arthralgia disease” in the category of “arthralgia disease” in TCM. Arthralgia, mostly caused by the feeling excesses of wind, cold, and dampness in muscles, bones, and meridians, manifests the pain, heavy, numbness, and adverse events of limb joints and muscles, whose pathogenesis is stagnation of qi and blood, and the fact the muscles and veins are not be nourished. In traditional Chinese medicine, the obstruction of qi and blood stasis is regarded as “impassability,” and the loss of nourishment of muscles and veins is regarded as “dystrophy.” Both impassability and dystrophy can lead to pain, numbness, and other symptoms. HXP mainly applies the method of promoting blood circulation and removing blood stasis to the main pathogenesis of impassability. Although modern medicine has no final conclusion on the etiology of KOA, most studies have reported that the disease is related to congenital factors, trauma, overweight, postmenopausal changes, lifestyle, work, and so on [26].

## 5. Conclusion

This study analyzes the treatment of KOA with HXP through NP, thus revealing that the specific mechanism of drug action may be mainly through effective components such as quercetin, luteolin, *β*-sitosterol, tanshinone IIA, dihydrotanshinolactone, and so on that achieve therapeutic effects by regulating relevant signals such as inflammatory response, apoptosis, and oxidation reaction, which provides direction and enlightenment for exploring the drug mechanism of HXP. At the same time, this study still has limitations. Firstly, as previously reported, signaling pathways can be cross-regulated with each other, and the pivotal signaling pathways of HXP in the treatment of KOA remain to be explored. Secondly, current research work mainly comes from bioinformatics analysis, thereby future research can be verified by in vitro and in vivo experiments. Finally, due to the limitations of current pharmacological techniques, it is impossible to determine the dose-response relationship between HXP and KOA.

## Figures and Tables

**Figure 1:** Wireless sensor network medical management system architecture.

**Figure 2:** Drug-disease common targets.

**Figure 3:** “Drug-component-target-disease” network model.

**Figure 4:** PPI network (left) and screening of core targets (right).

**Figure 5:** Bubble chart of the top 10 pathways of GO-BP analysis.

**Figure 6:** Bubble chart of the top 10 pathways of GO-BP analysis.

**Figure 7:** Bubble chart of the top 10 pathways of GO-CC analysis.

**Figure 8:** Bubble chart of the top 20 pathways of KEGG analysis.

**Table 1:** Some active ingredients of Huoluo Xiaoling Pill.

Mol ID	Chemical component	OB (%)	DL	Herb
MOL000006	Luteolin	36.16263	0.24552	Salvia miltiorrhiza
MOL002222	Sugiol	36.11353	0.27648	Salvia miltiorrhiza
MOL001942	Isoimperatorin	45.46425	0.22524	Salvia miltiorrhiza
MOL001771	Poriferast-5-en-3beta-ol	36.91391	0.75034	Salvia miltiorrhiza
MOL001601	1,2,5,6-Tetrahydrotanshinone	38.74539	0.35791	Salvia miltiorrhiza
MOL000569	Digallate	61.84862	0.25635	Salvia miltiorrhiza
MOL001659	Poriferasterol	43.82985	0.75596	Salvia miltiorrhiza
MOL001215	Tirucallol	42.11919	0.75003	Frankincense
MOL001241	O-acetyl-*α*-boswellic acid	42.72972	0.6963	Frankincense
MOL001243	3alpha-Hydroxy-olean-12-en-24-oic-acid	39.32421	0.7533	Frankincense
MOL001255	Boswellic acid	39.54759	0.75186	Frankincense
MOL001263	3-Oxo-tirucallic acid	42.85781	0.80503	Frankincense
MOL001001	Quercetin-3-O-*β*-D-glucuronide	30.65561	0.73645	Myrrh
MOL001002	Ellagic acid	43.06456	0.43417	Myrrh
MOL001004	Pelargonidin	37.98831	0.21204	Myrrh
MOL001006	Poriferasta-7,22E-dien-3beta-ol	42.97937	0.75555	Myrrh
MOL001009	Guggulsterol-VI	54.71797	0.43055	Myrrh
MOL000358	Beta-sitosterol	36.91	0.75	Angelica sinensis, myrrh
MOL000449	Stigmasterol	43.83	0.76	Angelica sinensis, myrrh

**Table 2:** 28 active ingredients in Huoluo Xiaoling Pill with connectivity not less than 10.

Active ingredients	Connectivity	Active ingredients	Connectivity
Quercetin	90	Danshenspiroketallactone	12
Luteolin	44	Dehydrotanshinone II A	11
Beta-sitosterol	32	Salviolone	11
Tanshinone IIa	24	Miltirone	11
Dihydrotanshinlactone	17	Deoxyneocryptotanshinone	11
Cryptotanshinone	17	1,2,5,6-Tetrahydrotanshinone	11
Stigmasterol	17	Przewaquinone C	11
Neocryptotanshinone II	14	Methylenetanshinquinone	11
Miltionone I	14	2-Isopropyl-8-methylphenanthrene-3,4-dione	11
Dan-shexinkum D	14	Pelargonidin	10
Ellagic acid	13	1-Methyl-8,9-dihydro-7H-naphtho[5,6-g]benzofuran-6,10,11-trione	10
Isotanshinone II	13	Epidanshenspiroketallactone	10
4-methylenemiltirone	13	3-Beta-hydroxymethyllenetanshiquinone	10
Isocryptotanshi-none	12	2-(4-Hydroxy-3-methoxyphenyl)-5-(3-hydroxypropyl)-7-methoxy-3-benzofurancarboxaldehyde	10

**Table 3:** Related pathways of Huoluo Xiaoling Pill in the treatment of knee osteoarthritis.

Channel number	*P* value	Pathway name	Participating gene
hsa04657	-30.549	IL-17 signaling pathway	CASP3, CASP8, CHUK, MAPK14, FOS, CXCL2, GSK3B, HSP90AA1, IFNG, IL1B, CXCL8, CXCL10, JUN, MMP1, MMP3, MMP9, NFKBIA, MAPK1, PTGS2, RELA, CCL2
hsa04668	-30.4926	TNF signaling pathway	AKT1, CASP3, CASP7, CASP8, CHUK, MAPK14, FOS, CXCL2, ICAM1, IL1B, CXCL10, JUN, MMP3, MMP9, NFKBIA, MAPK1, PTGS2, RELA, CCL2, SELE, VCAM1
hsa05169	-26.7835	Epstein-Barr virus infection	AKT1, BAX, CCND1, BCL2, CASP3, CASP8, CASP9, CDK, CDK4, CDKN1A, CHUK, MAPK14, E2F1, GSK3B, HSPB1, ICAM, IFNG, CXCL10, JUN, MDM2, MYC, NFKBIA, RELA, STAT1, STAT3, TP53
hsa04151	-22.7152	PI3K-Akt signaling pathway	AKT1, CCND1, BCL2, BCL2L1, CASP9, CDK4, CDKN1A, CHUK, EGFR, GSK3B, HSP90AA1, IL2, IL4R, ITGB3, MDM2, MET, MYC, NOS3, PRKCA, MAPK1, RELA, SPP1, TP53
hsa04210	-22.6584	Apoptosis	PARP1, AKT1, XIAP, BIRC5, BAX, BCL2, BCL2L1, CASP3, CASP7, CASP8, CASP9, CHUK, CTSD, FOS, JUN, NFKBIA, MAPK1, RELA, TP53
hsa04066	-21.2695	HIF-1 signaling pathway	AKT1, BCL2, CDKN1A, EGFR, ERBB2, F3, HIF1A, HK2, HMOX1, IFNG, NOS2, NOS3, SERPINE1, PRKCA, MAPK1, RELA, STAT3
hsa04115	-20.7752	p53 signaling pathway	BAX, CCND1, BCL2, BCL2L1, CASP3, CASP8, CASP9, CCNB1, CDK1, CDK4, CDKN1A, IGFBP3, MDM2, SERPINE1, TP53
hsa04064	-18.6693	NF-kappa B signaling pathway	PARP1, XIAP, BCL2, BCL2L1, CD40LG, CHUK, CXCL2, ICAM1, IL1B, CXCL8, NFKBIA, PLAU, PTGS2, RELA, VCAM1
hsa04620	-18.419	Toll-like receptor signaling pathway	AKT1, CASP8, CHUK, MAPK14, FOS, IL1B, CXCL8, CXCL1, JUN, NFKBIA, MAPK1, RELA, CXCL11, SPP1, STAT1
hsa04380	-16.9517	Osteoclast differentiation	AKT1, CALCR, CHUK, MAPK14, FOS, IFNG, IL1A, IL1B, ITGB3, JUN, NFKBIA, PPARG, MAPK1, RELA, STAT1
hsa04621	-16.412	NOD-like receptor signaling pathway	XIAP, BCL2, BCL2L1, CASP8, CHUK, MAPK14, CXCL2, HSP90AA1, IL1B, CXCL8, JUN, NFKBIA, MAPK1, RELA, CCL2, STAT1
hsa04010	-15.1529	MAPK signaling pathway	AKT1, CASP3, CHUK, MAPK14, EGFR, ERBB2, FOS, HSPB, IGF2, IL1A, IL1B, JUN, MET, MYC, PRKCA, MAPK1, RELA, TP53

## Data Availability

No data were used to support this study.
